# Diagnostic Accuracy and Usability of the ECG247 Smart Heart Sensor Compared to Conventional Holter Technology

**DOI:** 10.1155/2021/5230947

**Published:** 2021-11-02

**Authors:** Edvard Liljedahl Sandberg, Bjørnar Leangen Grenne, Trygve Berge, Jostein Grimsmo, Dan Atar, Sigrun Halvorsen, Rune Fensli, Jarle Jortveit

**Affiliations:** ^1^Sorlandet Hospital, Department of Cardiology, Arendal, Norway; ^2^Clinic of Cardiology, St. Olavs Hospital, Trondheim, Norway; ^3^Centre for Innovative Ultrasound Solutions and Department of Circulation and Medical Imaging, Norwegian University of Science and Technology, Trondheim, Norway; ^4^Vestre Viken Hospital Trust, Baerum Hospital, Department of Medical Research and Department of Internal Medicine, Rud, Norway; ^5^LHL-Hospital Gardermoen, Department of Cardiac Rehabilitation, Jessheim, Norway; ^6^Oslo University Hospital Ullevål, Department of Cardiology, Oslo, Norway; ^7^Institute of Clinical Medicine, University of Oslo, Oslo, Norway; ^8^Faculty of Engineering and Science, University of Agder, Grimstad, Norway

## Abstract

**Background:**

Heart rhythm disorders, especially atrial fibrillation (AF), are increasing global health challenges. Conventional diagnostic tools for assessment of rhythm disorders suffer from limited availability, limited test duration time, and usability challenges. There is also a need for out-of-hospital investigation of arrhythmias. Therefore, the Norwegian ECG247 Smart Heart Sensor has been developed to simplify the assessment of heart rhythm disorders. The current study aimed to evaluate the diagnostic accuracy and usability of the ECG247 Smart Heart Sensor compared to conventional Holter monitors.

**Methods:**

Parallel tests with ECG247 Smart Heart Sensor and a Holter monitor were performed in 151 consecutive patients referred for out-of-hospital long-term ECG recording at Sorlandet Hospital Arendal, Norway. All ECG data were automatically analysed by both systems and evaluated by hospital physicians. Participants were asked to complete a questionnaire scoring usability parameters after the test.

**Results:**

A total of 150 patients (62% men, age 54 (±17) years) completed the study. The ECG quality from both monitors was considered satisfactory for rhythm analysis in all patients. AF was identified in 9 (6%) patients during the period with parallel tests. The diagnostic accuracy for automatic AF detection was 95% (95% CI 91–98) for the ECG247 Smart Heart Sensor and 81% (95% CI 74–87) for the Holter system. The proportion of false-positive AF was 4% in tests analysed by the ECG247 algorithm and 16% in tests analysed by the Holter algorithm. Other arrhythmias were absent/rare. The system usability score was significantly better for ECG247 Smart Heart Sensor compared to traditional Holter technology (score 87.4 vs. 67.5, *p* < 0.001).

**Conclusions:**

The ECG247 Smart Heart Sensor showed at least comparable diagnostic accuracy for AF and improved usability compared to conventional Holter technology. ECG247 allows for prolonged monitoring and may improve detection of AF. This trial is registered with https://clinicaltrials.gov/ct2/show/NCT04700865.

## 1. Introduction

Heart rhythm disorders are common and may be associated with serious complications. A 12-lead electrocardiogram (ECG) is the gold standard for the diagnosis of rhythm disorders but can only provide a snapshot of the heart's electrical signals. Some frequent arrhythmias, such as atrial fibrillation (AF), may be missed due to its intermittent nature [1, 2]. AF is the most common cardiac rhythm disorder [2–6]. The most serious complication of AF is ischemic stroke [2, 7–9]. AF confers a 5-fold risk of stroke, and 20–30% of all strokes are attributed to this arrhythmia [8]. Anticoagulation therapy effectively reduces stroke risk in these patients [10]. However, up to one-third of AF cases are undiagnosed and untreated [11]. Consequently, there is a need for more effective diagnostic tools to identify AF.

Equipment for long-term ECG recording, often referred to as “Holter monitoring,” has been in clinical use since the 1950s [12]. A Holter monitor system requires a recording device coupled to at least three cables attached to electrodes on the chest. The system is bulky, difficult to conceal at work/public venues, has limited battery capacity (typically 1–3 days), and is sensitive to electric disturbances and movement artifacts. Today, several systems for long-term ECG monitoring are available, either with automatic detection or user-initiated recording of events. Home-based self-applied wearable ECG patch devices may facilitate the diagnosis of AF [13]. However, 1 of 4 patients is unable to activate an event recorder during a symptomatic period [14]. Implantable loop recorders provide an opportunity for prolonged continuous rhythm monitoring (months to years), but such devices require invasive procedures with high cost and potential risks. “Smart” watches with heart rate monitoring are usually based on the identification of arterial pressure waves. However, international guidelines require ECG documentation for the diagnosis of arrhythmias [2].

Approximately 1200 long-term ECG recordings are performed per 100, 000 inhabitants every year in Norway, and the number of procedures increased by 70% over the last ten years [15]. The procedures require specialized nurses and cardiologists and are time-consuming and resource intensive. Access to equipment may be limited, and long delays from onset of symptoms to examination may occur.

The ECG247 Smart Heart Sensor is a new digital clinical tool for out-of-hospital self-testing of cardiac arrhythmias and addresses most of the challenges with Holter systems, event recorders, and other devices. The concept consists of a wireless patch ECG sensor with real-time continuous (24 hours a day, 7 days a week), ECG analysis, a medical grade smartphone application, a secure medical back-end cloud service with automatic ECG analysis based on artificial intelligence algorithms, and a web portal.

The objectives of the present study were to evaluate the diagnostic accuracy and usability of ECG247 Smart Heart Sensor compared to conventional Holter monitoring.

## 2. Methods

### 2.1. Study Design

This prospective observational non-randomized diagnostic accuracy study was conducted and reported according to the STARD recommendations [16]. The study was conducted at Sorlandet Hospital Arendal, Norway, between September 2020 and March 2021.

### 2.2. Study Population

All consecutive patients ≥18 years of age referred for ordinary out-of-hospital long-term ECG recording at Sorlandet Hospital Arendal in the study period were screened for inclusion in the study regardless of indication or symptoms. Three study nurses at the cardiology outpatient's clinic were responsible for screening, inclusion, and obtaining informed consent. The exclusion criteria were lack of ability to cooperate, known skin allergies/sensitivity to components in the patch adhesives, and planned external cardioversion during the monitoring period.

### 2.3. Diagnostic Devices

The index tests were performed with ECG247 Smart Heart Sensor (Appsens, Lillesand, Norway). This wireless single-lead patch ECG monitoring device system consists of an electrode patch (battery included) with a lightweight reusable sensor, a smartphone application, a back-end cloud service, and a web portal (Figure 1). The water-resistant sensor attaches over the sternum (Figure 2) and continuously monitors the heart rhythm for up to 14 days without the need for charging. All ECG recordings are sent in real time from the ECG247 sensor using Bluetooth Low Energy (BLE) communication through a dedicated ECG247 application on the patient's mobile phone to a secure Microsoft Azure cloud storage solution with web-access for the user and for healthcare professionals (Figure 2). User authentication is provided by use of the Firebase Service, which gives a two-factor authentication required for access to sensitive medical information. All stored information is coded as Fast Health Interoperability Resources (FHIR). The ECG247 Smart Sensor continuously monitors the heart rhythm and has incorporated algorithms for real-time detections of arrhythmias. All arrhythmias are automatically uploaded to the secure cloud storage solution. A dedicated parameter defining the signal quality ensures high reliability of automatically detected arrythmias. For system reliability, a periodic recording of 1-minute ECG is detected every 30th minute and uploaded to the back-end services. Patient-initiated recordings can be activated by pressing a trigger button at the sensor. A flash memory in the sensor allows for saving of up to one hour of ECG recordings, in case of situations without BLE communication to the mobile phone.

All possible arrhythmias are immediately automatically re-analysed in the back-end service to verify or reject the sensor-detected events. The back-end analysing process consists of four distinct steps:

1. Analysing for detection of a beat (QRS complex) as an adaptive process where the typical beat waveform from the patient is analysed and updated every time a new periodic recording is uploaded. This process ensures reliable detection of a beat even in situations with variations in waveform (e.g., due to body position, physical activities, and skin humidity).
2. Identification of the correct beat type based on a machine-learning algorithm distinguishing between normal beats, supraventricular beats, ventricular beats, and artefacts. This algorithm has been developed in a supervised training process using a selection of manually annotated ECG recordings. The detected beat types and timing are stored as an annotation file, used both for the arrythmia analysing part but also used for correctly displaying the ECG recordings with the curve-plot having an overlay with beat annotations.
3. Analysing for arrhythmias or changes in regular rhythm as a state-machine process where the actual timing of changes in rhythms are important for verification of the arrhythmia. This process will also analyse for variations in R-R intervals to detect ectopic beats and AF. In addition, missing P-waves in front of R-waves are an important parameter for detection of AF. Changes in R-R intervals will also be used for detection of atrial flutter, low/high heart rate, supraventricular tachycardia, ventricular tachycardia, and pauses.
4. Analysing the ECG signal quality to avoid false triggering of arrhythmia detection due to artefacts, using a signal quality matrix filter.

This multiple-step algorithm method is implemented to verify real arrhythmias and to reduce the number of false-positive results. All R-R intervals are uploaded to the back-end services to generate a continuous graph of heart-rate variations during the investigation period. Main arrhythmia findings are automatically reported back to the user's phone application. All recordings are available in real time for both the user and for the healthcare professional after consent from the user in a web-based interface. The ECG247 Smart Heart Sensor system is designed according to the requirements given by the General Data Protection Regulation (GDPR) directive where the ownership to recorded information belongs to the user. The system is CE certified according to the EU Medical Device Directive (93/42/EEC).

A conventional Holter monitoring system (Medilog AR4 plus, Schiller, Baar, Switzerland) was used as reference standard in the study. The Medilog AR4 plus system consist of a recorder with five leads placed on the patient's chest with electrode patches. ECG data were transferred from the recorder to a stationary computer for analysis with Medilog Darwin software after the end of the test period.

### 2.4. Study Procedure

Outpatient parallel tests with ECG247 Smart Heart Sensor and Medilog AR4 plus Holter monitor were performed in all study patients after signed informed consent for study participation (Figure 3). Both systems were mounted by skilled study nurses and activated simultaneously. The participants were instructed to wear both systems for minimum twenty-four hours. All ECG data from the Medilog AR4 plus system were analysed according to the hospitals' standard routines by hospital physicians and a text report was prepared in the hospitals' medical records system. The original interpretation was accepted as reference standard. All ECG events from the ECG247 Smart Heart Sensor were manually analysed in the ECG247 web portal by two physicians. In case of doubt, a third physician (cardiologist) was consulted. Results from the index test were not available to the assessors of the reference standard. The occurrence and/or duration of supraventricular ectopic beats, supraventricular tachycardia (≥30 sec), atrial fibrillation (≥30 sec), atrial flutter (≥30 sec), ventricular ectopic beats, ventricular tachycardia (>4 beats), and pause (>4 sec) were recorded. Tests with insufficient data were excluded from the study.

All participants were asked to complete a digital questionnaire regarding baseline clinical information (gender, age, height, weight, previous cardiovascular disease, and use of anticoagulation therapy) and usability [17] 1–3 weeks after the test.

### 2.5. Outcomes

The primary outcome was the detection of the defined arrythmias recorded with the ECG247 Smart Heart Sensor System compared to the detection of the arrhythmias recorded with the Medilog AR4 Holter monitor (reference standard) in the period with parallel tests. The secondary outcome was the usability of both systems, measured by System Usability Score (SUS) [17].

### 2.6. Statistics

Continuous variables are presented as means ± SD (standard deviations) or medians (25th percentile, 75th percentile), and differences between groups were analysed using independent samples *t*-tests. Categorical variables are presented as numbers and percentages. Sensitivity, specificity, and accuracy are reported as percentages with Clopper–Pearson confidence intervals. Sample size calculation (*n* = 150) was based on an estimate of AF incidence in the study population (0.08), as well as an assumed sensitivity (0.97) with beta ≤0.2. A *p* value of <0.05 was regarded as statistically significant. The data were analysed using STATA version 16 (StataCorp LLC, College Station, TX, USA). Summary statistics for diagnostic tests and sample size estimation were conducted with the user-developed commands “diagt” and “diagsampsi” respectively.

### 2.7. Patient and Public Involvement

Three user representatives were consulted in the preparation of the study protocol, and feedback from participants was used to adjust the study procedure within the protocol frames.

### 2.8. Ethics

The Regional Committee for Medical and Health Research Ethics approved this study (REK 11479). All study participants have signed a written consent form.

## 3. Results

A total of 151 patients were included in the study at Sorlandet Hospital Arendal, Norway. One (1%) participant was excluded from further analysis due to technical problem with the use of the ECG247 system (private mobile phone without power). For all other tests, the ECG quality was considered satisfactory for rhythm analysis. A total of 93 (62%) participants were male, and mean age was 54 (±17) years. Self-reported medical history is presented in Table 1 (missing data in 31 (21%) participants).

Mean parallel ECG monitoring time was 33 (±22) hours. Some participants chose on their own initiative to use ECG247 Smart Heart Sensor longer due to, for example, weekends/holidays (closed outpatient clinic). Mean monitoring time with the ECG247 Smart Heart Sensor was 49 (±45) hours. The diagnostic accuracy of AF and ectopic beats in the time interval with parallel tests (33 (±22) hours) are presented in Table 2. AF was identified in 9 (6%) patients during the interval with parallel tests, and in another four patients after the Holter test was finished. AF appeared intermittently in six (46%) of these 13 patients. In one case, a short (<1 min) episode of AF was not detected by the ECG247 automatic arrhythmia detection algorithm. One AF episode (duration 5 min) was missed by the Holter algorithm and by the hospital physician. This AF episode was detected by the ECG247 Smart Heart Sensor. The proportion of false-positive tests identified as having AF was 4% (6 of 137) in tests analysed by the ECG247 algorithm and 16% (26 of 142) in tests analysed by the Holter algorithm. Other arrhythmias were absent or rare in the study population, and the diagnostic accuracy cannot be determined with reliability. Ectopic beats were present in the majority of the tests and were satisfactory identified by both systems.

The self-reported usability of the ECG247 Smart Heart Sensor System was in most situations significantly better compared to the conventional Holter system (Table 3). We found no differences between the systems regarding adverse events (Table 3).

## 4. Discussion

This diagnostic accuracy study included 151 parallel tests with ECG247 Smart Heart Sensor and a traditional Holter system for a mean duration of 33 hours and demonstrated at least comparable ability to detect frequent arrhythmias and significantly improved usability of the ECG247 Smart Heart Sensor compared to a conventional Holter system.

Ambulatory Holter monitors have been the most widely used clinical tool in the assessment of heart rhythm disorders over many decades. However, Holter monitors may be cumbersome to use and have limited test duration. Recent technological developments have enabled simplifications and improvements in the assessment of cardiac arrhythmias. The number of long-term ECG procedures is increasing [15]. There is no consensus in Europe regarding which patients should be referred for long-term ECG recording. There is a need for easy-to-use devices to assess cardiac arrhythmias outside hospitals and cardiology clinics.

A single-lead ECG from a patch sensor may be more difficult to analyse for an automatic algorithm and to interpret by a physician compared to a 3-lead ECG from a Holter system. The number of leads is less important for the interpretation of narrow QRS complex arrhythmias like AF. The diagnostic accuracy for AF by the ECG247 Smart Heart Sensor was comparable to the Holter system in the parallel observation period of 33 hours. The number of false-positive AF was low in tests performed by ECG247 Smart Heart Sensor (4%) compared to tests performed by the Holter system (16%). Multiple-lead recordings may improve detection of arrhythmias characterized by a shift in the electrical axis and/or altered QRS morphology (e.g., ventricular tachycardia). The number of ventricular arrhythmias observed in this study was too low to define the diagnostic accuracy for such arrhythmias.

Many patients in this study found the ambulatory Holter monitor uncomfortable to wear during daily activities. Similar findings have been reported from other studies [18, 19]. The ECG247 Smart Heart Sensor interferes less with daily activities (e.g., sleeping, exercising, or showering). The device can easily be used during exercise and sports and allows for longer monitoring periods. Prolonged ECG monitoring increases the diagnostic yield of ECG tests [20]. We observed an indication for this, as four additional patients had AF detected after completing the Holter test. Optimal observation time has not been clarified, but previous studies indicate that up to 7 days is desirable [20]. Hence, the ECG247 Smart Heart Sensor may increase detection rate of AF and other arrhythmias.

The European Society of Cardiology recommends screening for AF in patients at increased risk of stroke [2]. Long-term continuous ECG recording increases the likelihood of detecting paroxysmal AF compared to intermittent ECG recording [21]. However, there is currently limited long-term continuous ECG recording equipment available that is suitable, affordable, and sufficiently easy to use for screening purposes [22]. The ECG247 Smart Heart Sensor may represent an opportunity for AF screening in large populations.

The coronavirus disease 2019 (COVID-19) pandemic demonstrates the need for out-of-hospital self-testing diagnostic tools. The ECG247 Smart Heart Sensor enables transition of the assessment of arrhythmias from the hospitals to the patient's home and from the specialist health service to the primary health service. The sensor can be mailed directly to the user and self-applied, and all ECG recordings are available in real time for healthcare professionals.

The current study has several limitations. It was a single-center study, based on relatively few patients and selected health care professionals with in-depth knowledge of both long-term ECG monitoring systems. The study enrolled patients referred for long-term ECG monitoring without any evaluation of the risk of arrhythmias. Consequently, the absolute number of arrhythmias was low. The participants' possible enthusiasm for testing new technology may also represent a possible bias.

Despite these limitations, we conclude that the ECG247 Smart Heart Sensor showed comparable diagnostic accuracy and improved usability compared to conventional Holter technology in this study. However, a larger study is needed to determine the diagnostic utility of the system.

## Figures and Tables

**Figure 1:** The ECG247 Smart Heart Sensor system: sensor with real-time arrhythmia detection, smartphone application, back-end cloud service with postprocessing arrhythmia analyser, and web portal.

**Figure 2:** The ECG247 Smart Heart Sensor placed over the sternum, screenshots from the ECG247 mobile application, and a screenshot from the ECG247 web portal for healthcare professionals.

**Figure 3:** Parallel tests with ECG247 Smart Heart Sensor and Medilog AR4 Holter monitor.

**Table 1:** Self-reported medical history in patients with long-term ECG recording, *n* = 120 (missing self-reported health data in 31 patients).

	*n* = 120
Permanent atrial fibrillation, *n* (%)	6 (5)
Paroxysmal atrial fibrillation, *n* (%)	34 (28)
Diabetes, *n* (%)	10 (8)

Previous coronary heart disease	
Myocardial infarction, *n* (%)	10 (8)
Percutaneous coronary intervention, *n* (%)	19 (16)
Coronary artery bypass grafting, *n* (%)	1 (1)

Previous stroke, *n* (%)	17 (14)
History of heart failure, *n* (%)	3 (3)
Anticoagulation therapy, *n* (%)	42 (35)

**Table 2:** Diagnostic evaluation of the arrhythmia detection in parallel tests with ECG247 Smart Heart Sensor and conventional Holter technology.

Arrhythmia and ectopic beats, *n* = 150	Diagnostic evaluation	ECG247 algorithm, 95% CI	ECG247 algorithm and physician review, 95% CI	Holter algorithm, 95% CI	Holter algorithm and physician review, 95% CI
Atrial fibrillation	Sensitivity	8/9 = 89% (52–100)	9/9 = 100% (66–100)	7/9 = 78% (40–97)	8/9 = 89% (52–100)
	Specificity	135/141 = 96% (91–98)	141/141 = 100% (97–100)	115/141 = 82% (74–88)	141/141 = 100% (97–100)
	Positive predictive value	57% (37–75)	100%	21% (14–31)	100%
	Negative predictive value	99% (96–100)	100%	98% (94–99)	99% (96–100)
	Diagnostic accuracy	95% (91–98)	100% (98–100)	81% (74–87)	99% (96–100)

Ventricular ectopic beats	Sensitivity	114/122 = 93% (87–97)	114/122 = 93% (87–97)	114/122 = 93% (88–97)	118/122 = 97% (92–99)
	Specificity	8/28 = 29% (13–49)	28/28 = 100% (88–100)	16/28 = 57% (37–76)	28/28 = 100% (88–100)
	Positive predictive value	85% (82–88)	100%	90% (86–94)	100%
	Negative predictive value	50% (29–71)	78% (64–87)	67% (49–81)	88% (73–95)
	Diagnostic accuracy	81% (74–87)	95% (90–98)	87% (80–92)	97% (93–99)

Supraventricular ectopic beats	Sensitivity	130/135 = 96% (92–99)	130/135 = 96% (92–99)	131/135 = 97% (93–99)	131/135 = 97% (93–99)
	Specificity	7/15 = 47% (21–73)	15/15 = 100% (78–100)	9/15 = 60% (32–84)	15/15 = 100% (78–100)
	Positive predictive value	94% (91–96)	100%	96% (92–98)	100%
	Negative predictive value	58% (34–79)	75% (56–88)	69% (44–87)	79% (59–91)
	Diagnostic accuracy	91% (86–95)	97% (92–99)	93% (88–97)	97% (93–99)

**Table 3:** Usability of ECG247 versus Holter technology in patients with long-term ECG recording, *n* = 120 (missing data in 31 patients).

	ECG247	Holter technology	Diff.	*p*
*Mean usability score in different situations (SD)* ^1^				
Showering	2.8 (3.0)	7.0 (3.7)	4.2	<0.001
Training	1.6 (1.4)	4.6 (3.3)	3.0	<0.001
Sleeping	1.6 (1.2)	4.2 (2.7)	2.6	<0.001
Physical activity	1.2 (0.5)	2.9 (2.3)	1.7	<0.001
At work	1.1 (0.5)	2.4 (2.0)	1.3	<0.001
WC	1.0 (0.1)	2.2 (1.9)	1.2	<0.001
Social relations	1.1 (0.3)	2.2 (2.0)	1.1	<0.001
Eating	1.1 (0.4)	1.5 (1.1)	0.4	<0.001

*Adverse events score* ^2^				
Itching	2.8 (2.5)	3.0 (2.7)	0.2	0.49
Erythema	2.9 (2.7)	3.1 (2.8)	0.2	0.59

System usability score^3^	87.4 (1.4)	67.5 (1.8)	19.9	<0.001

^1^Usability score: 1 (excellent)–10 (very poor). ^2^Adverse event score: 1 (no problem)–10 (not acceptable). ^3^System usability score: 0–100, >68 acceptable.

## Data Availability

The data that support the findings of this study are available on request from the corresponding author (ES).
